# The Impact of a Knowledge Discovery-Based Psychoanalytic Intervention in the Treatment of Tuberculosis in University Students with Different Doses of Isoniazid

**DOI:** 10.1155/2022/5610469

**Published:** 2022-03-21

**Authors:** Zhihui Xia, Youping Tan, Yumei Yang

**Affiliations:** ^1^North China Electric Power University Hospital, Health Care Department, Changping, Beijing 102206, China; ^2^Department of Hematology, Guangdong Second People's Hospital, Guangzhou, Guangdong 510310, China; ^3^Medical and Nursing College, Wuhan Railway Vocational and Technical College, Wuhan, Hubei 430205, China

## Abstract

Tuberculosis (TB) is an infectious disease that poses a serious threat to the health of the population in China, and TB outbreaks in universities have aroused great concern in society. Psychological emotions have a large impact on the academic lives of university students, and nowadays it is not only labour-intensive but also slow to monitor and analyse and deal with the psychology of university students' daily lives in a uniform manner. If psychological problems are not detected and given feedback in a timely manner, they can have a series of negative effects on the individual university student. In this paper, we apply the Bi-LSTM model and the CNN model neural network algorithm to learn the text data, and finally have 95.55% and 90.03% accuracy in the sentiment analysis experiment, respectively, which provides a feasible solution to solve the batch rapid analysis of the psychological changes reflected in the daily text of university students. Risk communication for TB emergencies should emphasize public participation, timely release of information about the epidemic, and good monitoring of public opinion.

## 1. Introduction

Tuberculosis (TB) is a chronic respiratory infectious disease. It ranks second in China in terms of the incidence of infectious diseases and has become one of the major diseases that seriously affect the health of the population [1]. In recent years, the prevention and control of *tuberculosis* in schools has attracted a great deal of attention from all sectors of society, especially from university students, who have a high incidence of *tuberculosis* and the potential for outbreaks due to factors such as relocation, changes in the social environment, and increased pressure from studies and employment [2].

The important role of risk communication [3] in emergency situations has gradually been recognized by the society in recent years. Knowledge discovery is included in the Ministry of Health document: “Strengthen risk communication and crisis communication. The importance of risk communication in daily work and information dissemination in the management of emergencies should be fully recognized” [4]. The purpose and significance of risk communication in the management of university *tuberculosis* outbreaks are as follows: in the event of a public health emergency, focusing on the reactions of all parties to the risk of disease and disseminating strategic measures for prevention and control by government or health management departments [5]. The most important purpose of risk communication is to build trust between the parties involved in an epidemic. This is where risk communication differs from general mass communication; the establishment and strength of trust is mutually dependent on the success or failure of risk communication and ultimately plays an important role in the development of effective risk decision-making, risk management, and risk early warning [6].

In the case of university TB outbreaks, the role of risk communication is to enable universities, education authorities, health authorities, students, staff, parents, the media, and the public to understand the facts of the incident, form a common understanding, establish a relationship of mutual trust, and work together to overcome risks. Risk communication is an integral part of the management of a TB outbreak and is important for the effectiveness of the management measures [7].

Identify the stakeholders in the management of a TB outbreak at the university so as to define the scope for the selection of communication targets. Risk communication can be divided into the following: internal communication, media communication, and public communication [8–10]. Internal communication is mainly aimed at medical and nursing staff, disease prevention and control staff, and health administration staff. Health administrative departments are responsible for organising internal communication, clarifying their respective responsibilities and scope of work in epidemic management, and coordinating conflicts, while medical workers should make full use of their professional advantages to audit the accuracy of the information released [11].

Sentiment analysis [12], also known as sentimental disposition analysis, is a direction of natural language processing, which is the process of analysing, generalizing, and reasoning through subjective texts with emotional overtones. In recent years, the development of the Internet has brought a large amount of data, making the advantages of natural language processing in terms of extracting features, classification speed, etc., increasingly significant. It is widely used in areas such as bulk user prediction and opinion induction. Deep learning is a type of machine learning that analyses and predicts data by using multiple nonlinear transformation structures to abstract the data at a higher order from large amounts of data. Convolutional neural network (CNN) [13] has been improved from image recognition and speech recognition to natural language processing in recent years and has achieved great success in processing short segments of speech. Gradient disappearance is based on bidirectional processing that can be analysed in conjunction with the context. In this paper, we compare and analyse the advantages and disadvantages of Bi-LSTM models and CNN models, and find a number of feasible features [14].

## 2. Theoretical Background

The dissemination of health information in advance will not only give all parties at the university sufficient time to make psychological adjustments in the event of an epidemic, but will also prepare public opinion and lay the groundwork for prevention and control of the epidemic in advance [15]. A good system of morning and afternoon check-ups and information sharing on the management of student sick leave registration should be implemented, and information between the universities should be shared.

The establishment of daily communication channels and mechanisms for health information between doctors and class teachers, between class teachers and class cadres, and between department heads and university leaders also has a positive effect on the early detection and reporting of epidemics, while the development and rehearsal of emergency plans should also incorporate risk communication to lay a good foundation for public health emergency work [16].

After a university *tuberculosis* outbreak, risk communication should be closely focused on the actual aspects and specific measures of university *tuberculosis* outbreak management, in line with the implementation of various prevention and control measures [17]. The development of strategies for risk communication in university TB epidemics; the timely release of epidemic information in university TB epidemic management; risk communication should also do a good job of monitoring public opinion and using monitoring data as an important basis for strategy development; paying attention to the amount of information released and the frequency of information release; and risk communication should make use of all possible means of communication. The epidemic management always also needs to deal with the following two contradictions: first, dealing with the timeliness and accuracy of risk; and second, the contradiction between timeliness and accuracy of information dissemination. On the basis of timeliness, acknowledging the uncertainty of the development of the epidemic, efforts should be made to ensure the relative accuracy of information in order to avoid filling the information vacuum before the release of “official” information with misinformation on the one hand, and to leave room for future policy adjustments on the other [18].

## 3. Related Technologies

### 3.1. Word Vectors

Computer deep learning requires the text to be segmented and then transformed into a vector form. One-hot representation [19] represents a word as a vector of length equal to the size of the lexicon, with only one padded 1 on the vector, indicating the position in the lexicon, and all the rest padded 0. The Euclidean distance between each vector is √2. One-hot encoding is simple to set up, but results in slow training due to an explosion of parameters in the text. One-hot encoding is simple to set up, but results in an explosion of parameters in the text, which leads to slow training. Moreover, discrete representation cannot represent the relationship between two words, and each word is isolated from each other, resulting in the inability to distinguish between synonyms in natural language processing work [20].

### 3.2. Neural Network Models

Neural networks are machine learning algorithms that mimic the human brain and are highly expressive and good fits for data. By setting up multiple hidden layers, it can automatically learn from the bottom features of the training data to the top features, as shown in Figure 1 [21]. The expression of the neural network is as follows:

(1) $$\begin{array}{c} y=NN\left(x\right), \end{array}$$

where *x* is the input vector, and *y* is the task-related output.

## 4. Models in This Paper

The model will be trained by the above process to obtain the final neural network parameters suitable for the needs of this paper. (1) The text is transformed into one-hot encoding using Python's Jieba library; (2) the one-hot encoding is pretrained by word2vec and transformed into word embedding vectors as input to the neural network; (3) the model is trained by Bi-LSTM network or CNN model to obtain; and (4) multiplying by fully connected layers and multiclassifying by software function to obtain sentiment tendency results. In this paper, we summarize the comparison between Bi-LSTM and CNN models on the basis of this process, as shown in Figure 2.

## 5. Case Studies

### 5.1. Information

In this study, 85 patients with TBM with mild anxiety symptoms admitted to our hospital between August 2016 and August 2019 were selected as the main study subjects. Inclusion criteria were as follows: patients with meningeal enhancement on cranial CT or MRI, confirmed by cerebrospinal fluid (CSF) and clinical features, and meeting the diagnostic criteria for tuberculous meningitis in the 2003 edition of Tuberculosis [22]; with a mean SAS score of 54.67 ± 1.85 and a mean SDS score of 57.31 ± 1.60. 42 patients had different degrees of headache, 42 patients had increased cranial pressure, and 40 patients had meningeal irritation.

Patients in both groups were treated according to the WHO recommended antituberculosis quadruple regimen and given oral paroxetine tablets at 20 mg/d, which could be increased to 40 mg/d depending on the patient's condition. INH 200 mg + dexamethasone 5 mg intrathecally in the low-dose group and INH 200 mg + dexamethasone 5 mg in the high-dose group.

Intrathecal injections were administered at the time of infusion. Once a week, the number of injections was adjusted according to the level of cerebrospinal fluid biochemical parameters. Both groups were treated continuously for 3 months, and the treatment effects were compared.

According to the modern hospital practice, the effect of TBM treatment in this study was evaluated [23, 24]. Clinical signs and symptoms of TBM improve slightly, and CSF levels improve to some extent on cerebrospinal fluid examination, but are not satisfactory.

## 6. Results

At the end of 3 months of treatment, the clinical efficacy was evaluated according to the “Modern Hospital Treatment Practice.” 18 cases were clinically cured, 12 cases were effective, 7 cases were effective, and 5 cases were ineffective in the small-dose group; 21 cases were clinically cured, 15 cases were effective, 6 cases were effective, and 1 case was ineffective in the high-dose group. The total effective rate of the high-dose group was 97.67% (42/43), higher than that of the small-dose group, which was 88.10% (37/42) (*χ*2 = 0.9417, *P* < 0.05).

### 6.1. Comparison of SAS and SDS Scores between the Two Groups

After treatment, the SAS and SDS scores of patients in both groups were significantly lower than before, and the scores of patients in the high-dose group were significantly lower than those in the low-dose group (*P* < 0.05), as shown in Table 1.

Before treatment, there was no statistically significant difference in the cell count, chloride level, protein content, and glucose of the cerebrospinal fluid between the two groups (*P* > 0.05). After treatment, the cell count, chloride level, protein content, and glucose in both groups improved significantly compared with before, and the improvement in biochemical indexes was better in the high-dose group than in the low-dose group (*P* < 0.05), as shown in Table 2.

During the treatment period, one case each of electrolyte abnormality, mild liver injury, and mild peripheral neuritis occurred in the low-dose group; two cases of electrolyte abnormality, and one case of mild hearing impairment, one case each of mild peripheral neuritis and liver injury occurred in the high-dose group. The incidence of drug-related adverse reactions was 9.30% in the high-dose group and 7.14% in the low-dose group, with no statistically significant difference (*x*^2^  = 16910, *P* > 0.05).

## 7. Experiment

### 7.1. Experimental Setup

In this paper, the dataset is obtained from the public dataset of IMDB, with 50,000 items and a positive to negative sample ratio of 1 : 1. After preprocessing, it is divided into a training set of 20,000 items, a development set of 5,000 items, and a test set of 25,000 items. The training set was used to train the neural network model. Then, the data from the development set were used for model selection and parameter tuning, and finally, the test set was used to evaluate the generalisation ability of the model [25, 26].

The experimental parameters directly affect the experimental results of the models. In this paper, we compare the number of hidden layers, the optimisation function, the dropout, filter size, and filter number of the CNN for different Bi-LSTMs after repeated experiments to arrive at the optimal initial parameters for the two models.  Table 3 shows the parameters of the Bi-LSTM, and Table 4 shows the parameters of the CNN.

### 7.2. Experimental Results

This paper not only compares the accuracy of the Bi-LSTM and CNN models, but also trains the classical RNN model and the LSTM model to help analyse the strengths and weaknesses of the models for the application in this paper. The experimental results are shown in Table 5.

It can be seen that the Bi-LSTM has a better result than the LSTM in terms of contextual analysis and a 5.52% higher accuracy than the CNN model. The prediction is that CNN does not have a high accuracy rate in the analysis of long passages due to the varying sentence lengths in the dataset. The LSTM is better than the RNN but still cannot make accurate predictions due to the inability to incorporate the following content. The results of this paper indirectly suggest that the daily textual expressions of university students are scattered among the segments, which is likely to be missed if manual analysis is conducted. The 95.55% accuracy of Bi-LSTM is good enough for batch text processing [27, 28].

This paper presents a comparative study of the performances of Bi-LSTM models, CNN models, and traditional neural network models to solve the psychological problem of batch analysis of university students. A feasible solution is proposed for the back analysis of daily texts of university students. For daily sentiment analysis, this paper starts with the natural language processing aspect of text, but can also be evaluated comprehensively with various aspects such as image and speech processing. In the future, the image literacy algorithm will be invoked to filter out some suitable computational nodes and then sort them so as to select an optimal node host, as showed in Figure 3 Different sentiment analysis effects.

The performance test is based on the response time and throughput of creating one virtual machine instance and the maximum number of virtual machines that can be successfully created by a single server, as shown in Figure 4.

In the current environment, up to 32 virtual machines can be created; it takes 320s to create the first instance of a virtual machine, and thereafter about 15 to 20 s to create virtual machines of the same image, as shown in Figure 5 for mental comfort when creating virtual machines in bulk. The first virtual machine takes longer as it needs to be found and copied when it is created. After the first VM is created, VMs are created quickly and the time remains relatively constant [29].

## 8. Discussion

Modern medicine has confirmed [30] that TBM is highly infectious, disabling, and fatal, and that if intervention is not timely during the acute phase, it can easily turn into chronic meningoencephalitis, with pathological changes such as basal ganglia exudate and hydrocephalus causing lesions to be deposited at the base of the skull and eventually causing permanent neurological complications, especially when symptoms of parenchymal damage appear at 4–8 weeks of onset, manifesting as mental depression, apathy, indifference, delirium, or delusions. Delirium or delusions, and even varying degrees of anxiety, depression, lethargy, confusion, or partial epilepsy. Therefore, treatment of patients with TB meningitis with anxiety and depression should be initiated early with antituberculosis and antianxiety and depression treatment.

Isoniazid (INH), a commonly used antituberculosis drug, can rapidly penetrate the blood-brain barrier and penetrate into the cerebrospinal fluid regardless of whether the patient has meningitis. Modern pharmacogenetics studies have shown that high concentrations of INH can kill *Mycobacterium tuberculosis* in the reproductive phase and that it is equally effective against *Mycobacterium tuberculosis* in the stationary phase if the blood concentration is increased or the contact time with the bacteria is prolonged. In this study, the total effective rate was 97.67% (42/43) in the high-dose group, which was higher than the total effective rate of 88.10% (37/42) in the low-dose group (*P* < 0.05). It was suggested that the INH 200 mg + dexamethasone 5 mg regimen was more effective than the INH 100 mg + dexamethasone 5 mg intrathecal injection, which was generally consistent with the results of [25] studies.

The mental status of patients with TBM is closely related to *tuberculosis* intoxication, meningeal irritation, increased cranial pressure, cerebral nerve injury, and brain parenchymal damage. INH was considered the first antidepressant, but was withdrawn from the market because of its high hepatotoxicity [27]. In this study, both treatment regimens reduced the SAS and SDS scores of patients after treatment, but the high-dose group reduced the SAS and SDS scores to a greater extent than the control group (*P* < 0.05), suggesting that oral paroxetine tablets combined with intrathecal INH could significantly improve the patients' mental status.

In conclusion, INH 200 mg intrathecal injection combined with paroxetine tablets significantly improved the mental status, cerebrospinal fluid cell count, chloride level, protein level, and glucose level in patients with TBM with anxiety and depression, which is important in improving the prognosis.

## 9. Conclusion

The university will play an important role in the management of the *tuberculosis* epidemic. With the substantial increase in computer computing power, deep learning natural language processing can help people analyse and solve previously unsolvable problems in productive life. Psychological emotions have a large impact on the academic lives of university students. Nowadays, unified monitoring and analysis of the psychology of university students' daily lives is not only labour-intensive but also slow. This paper applies the Bi-LSTM model and CNN model neural network algorithm to learn text data, and finally has a 95.55% and 90.03% accuracy rate, respectively, in the sentiment analysis experiment, which provides a feasible solution to solve the batch rapid analysis of the psychological changes reflected in the daily text of university students.

## Figures and Tables

**Figure 1:** Skip-gram model.

**Figure 2:** Flowchart of our model.

**Figure 3:** Effect of different sentiment analysis.

**Figure 4:** The effect of psychological comfort at different nodes.

**Figure 5:** Optimised psychological comfort effect.

**Table 1:** Comparison of SAS and SDS scores before and after treatment between the two groups ($\bar{x}\pm s$, scores).

Group	Number of cases	SAS score		SDS score	
		Before treatment	After treatment	Before treatment	After treatment
Low-dose group	42	54.67 ± 1.85	44.92 ± 1.67	57.31 ± 1.6	43.27 ± 1.55
High-dose group	43	54.62 ± 1.81	39.33 ± 1.65	57.29 ± 1.59	36.81 ± 1.56

**Table 2:** Comparison of cerebrospinal fluid biochemical indicators between the two groups before and after treatment $\left(\bar{x}\pm s\right)$.

Group	Number of cases	Cell count (10^6^/L)		Chloride level (mmol/L)		Protein content (g/L)		Glucose (mmol/L)	
		Before treatment	After treatment	Before treatment	After treatment	Before treatment	After treatment	Before treatment	After treatment
Low-dose group	42	436.25 ± 55.19	177.49 ± 39.92	97.71 ± 10.31	102.99 ± 10.54	6.65 ± 1.27	4.88 ± 1.19	1.11 ± 0.25	1.49 ± 0.28
High-dose group	43	436.33 ± 55.26	115.07 ± 36.22	98.75 ± 5.66	97.78 ± 10.29	116.43 ± 10.63	6.67 ± 1.28	1.12 ± 0.24	1.94 ± 0.29

**Table 3:** Bi-LSTM parameters.

Parameter	Value	Parameter	Value
Batch size	64	Learning rate	0.001
Unit num	32	Loss function	Cross entropy
Bi-LSTM	32	Optimization function	Random gradient descent
Epoch	6	Word vector dimension	256
Activation function	LeakyReLU		

**Table 4:** CNN parameters.

Parameter	Value	Parameter	Value
Filter size	3*∗*3	Dropout rate	0.5
Number of filters	100	Epoch	6
Activation function	ReLU	L2	3
Pooling method	Max	Word vector dimension	256

**Table 5:** Comparison of experimental results.

Model	Acc
Bi-LSTM	95.55
CNN	90.03
LSTM	85.07
RNN	81.33

## Data Availability

The data underlying the results presented in the study are available within the manuscript.
